# Artificial Intelligence and Deep Learning Assisted Rapid Diagnosis of COVID-19 from Chest Radiographical Images: A Survey

**DOI:** 10.1155/2022/1306664

**Published:** 2022-10-12

**Authors:** Deepak Sinwar, Vijaypal Singh Dhaka, Biniyam Alemu Tesfaye, Ghanshyam Raghuwanshi, Ashish Kumar, Sunil Kr. Maakar, Sanjay Agrawal

**Affiliations:** ^1^Department of Computer and Communication Engineering, Manipal University Jaipur, Jaipur, India; ^2^Department of Computer Science, College of Informatics, Bule Hora University, Bule Hora, Ethiopia; ^3^Department of Mathematics and Statistics, Manipal University Jaipur, Jaipur, India; ^4^School of Computing Science & Engineering, Galgotias University, Greater Noida, India; ^5^Department of Electrical Engineering, Rajkiya Engineering College, Akbarpur, Ambedkar Nagar, India

## Abstract

Artificial Intelligence (AI) has been applied successfully in many real-life domains for solving complex problems. With the invention of Machine Learning (ML) paradigms, it becomes convenient for researchers to predict the outcome based on past data. Nowadays, ML is acting as the biggest weapon against the COVID-19 pandemic by detecting symptomatic cases at an early stage and warning people about its futuristic effects. It is observed that COVID-19 has blown out globally so much in a short period because of the shortage of testing facilities and delays in test reports. To address this challenge, AI can be effectively applied to produce fast as well as cost-effective solutions. Plenty of researchers come up with AI-based solutions for preliminary diagnosis using chest CT Images, respiratory sound analysis, voice analysis of symptomatic persons with asymptomatic ones, and so forth. Some AI-based applications claim good accuracy in predicting the chances of being COVID-19-positive. Within a short period, plenty of research work is published regarding the identification of COVID-19. This paper has carefully examined and presented a comprehensive survey of more than 110 papers that came from various reputed sources, that is, Springer, IEEE, Elsevier, MDPI, arXiv, and medRxiv. Most of the papers selected for this survey presented candid work to detect and classify COVID-19, using deep-learning-based models from chest X-Rays and CT scan images. We hope that this survey covers most of the work and provides insights to the research community in proposing efficient as well as accurate solutions for fighting the pandemic.

## 1. Introduction

World Health Organization (WHO) announced COVID-19 (COrona VIrus Disease-2019) on February 11, 2020, as the name of a new disease which is caused by the 2019 novel coronavirus (2019-nCoV). Coronavirus is among the large family of Middle East Respiratory Syndrome (MERS-CoV) and severe acute respiratory syndrome (SARS-CoV) that causes diseases from cold infections. It is one of the newest viruses that were not discovered previously in humans. Typical signs of infection include cough, sore throat, fever, fatigue, headache, muscle pain, and breath shortness. COVID-19 pandemic is attributable to its property of respiratory transmission from one person to another, which causes the rapid spread of the disease. Wuhan in China reported the first case of COVID-19 in December 2019. WHO announced the coronavirus outbreak as a public health emergency of international concern on January 30, 2020, because it has affected the whole globe physically, socially, economically, and in many other areas. Its impact forces most of the affected countries to announce and implement a complete lockdown in the country. Since the first case in December 2019, the total number of infected people has reached more than 568 million as of Jul 20, 2022, including 6 million deaths. There are two main reasons for these numbers, namely, fast-spreading nature of 2019-nCov and late arrival of symptoms after getting infected. People come to know after 10–14 days that they have been infected with this virus. As a result, during this period, thousands of people get infected from that affected person. The deficiency of facilities, namely, rapid identification of disease, laboratory facilities, isolation facilities, doctors, other staff, Personal Protective Equipment (PPE) kits, and medicines, increases the risk of viral transmission. In general, we can say that the spreading rate of 2019-nCov is exponential. Jiang et al. [1] have also modeled the shape of such epidemics to be exponential. The total infected cases of countries are getting double in just a few days because the characteristics of 2019-nCov are not fully recognized yet. It is hard to discover the positive cases at an early stage. That is why it is of utmost importance to detect COVID-19 at an early stage to prevent its spreading. Governments are continuously issuing precautionary guidelines to the citizens for seeking cooperation in this regard. They used to advise citizens to follow social distancing and suspended industrial/school/office activities. It is the only way by which one can stay safer from getting infected. The situation of such a mysterious virus seems to be out of control as of now.

Many researchers are trying to devise mechanisms to investigate faster, reliable, and accurate detection of the disease. In general, we can classify all these techniques into two categories, namely, clinical examinations in the laboratory and other mechanisms (applying computational intelligence techniques, i.e., AI, ML, DL, and statistics). The goal of all these techniques has a single destiny, that is, to screen COVID-19 at an early stage. From the beginning, the validity of disease detection mainly depends on the earlier one, that is, clinical examinations. One of the famous techniques of this kind is Reverse Transcription-Polymerase Chain Reaction (RT-PCR). As compared to RT-PCR, computer-based detection can also help pathologists in a significant way because RT-PCR is a time-consuming investigation. It is sure that AI will not stop this pandemic but it can track and respond to the global emergency.

The performance of these techniques heavily depends on the availability of data. They perform better when the size of data is relatively large. Here the authors have focused more on AI-enabled technologies for predicting or handling the disease outbreaks. Many researchers have claimed to detect COVID-19 from chest X-ray images using deep learning techniques. However, the size of their datasets is not so large as it needs to be. Therefore, this study aims to present a comprehensive survey of work done by several researchers in diagnosing COVID-19 from chest radiographic images, that is, CT samples and X-ray images. The papers reviewed in this study are obtained from reputed sources, for example, ScienceDirect, Springer, MDPI, The Lancet, medRxiv, and arXiv preprints. Only specific studies related to deep learning models for early diagnosis of COVID-19 from radiographic images have been considered after applying several filters. The main contributions of this survey are highlighted as follows:

1. Comprehensive discussion of some AI-based solutions (mobile Apps, CT software, knowledge-based systems, etc.) for dealing with the COVID-19 pandemic.
2. In-depth review as well as the illustration of architectures of several deep-learning-based approaches (convolutional neural networks) for rapid diagnosis of COVID-19 from chest CT scans and X-ray images.
3. Comparative study of classification accuracies of several deep learning models in classifying COVID-19 from other types of pneumonia from CT scans and X-ray images.
4. Brief discussion of several computational approaches for analyzing and predicting the COVID-19 pandemic trends.
5. Presenting several imaging datasets for encouraging COVID-19 research.
6. Highlighting the pros and cons of deep-learning-based approaches for COVID-19 along with pointing out several open research issues.

The rest of the paper is structured as follows.  Section 2 discusses the importance of Artificial Intelligence in COVID-19 by presenting a few AI-based solutions that can play a vital role in coping with the COVID-19 outbreak. Deep-learning-based approaches for the identification of COVID-19 from the chest CT scan and X-ray images are briefed in Section 3 and Section 4, respectively.  Section 5 highlights some contributions of computational approaches other than deep learning for coping with the COVID-19 pandemic. Some COVID-19 public imaging datasets for performing the deep-learning-based research are presented in Section 6. A brief discussion of the pros and cons of using deep learning in solving real-life problems is presented in Section 7. Finally, Section 8 concludes the study with future directions.

## 2. AI-Enabled Solutions for COVID-19

AI-based automated disease detections are becoming more popular nowadays. There are several advantages of detecting COVID-19 using AI-based techniques, namely, faster detection, fewer chances of being affected while collecting and testing samples, cost-effectiveness, portability, and no worries about the availability of testing kits. During the initial stages of the COVID-19 outbreak, only a few repositories with limited COVID-19 patients' images were available. However, nowadays, there are many accessible progressive repositories to help the research community deploy and test their deep-learning-based models. Some sample X-ray and CT scan images of COVID-19-affected lungs are shown in Figures 1(a) and 1(b), respectively.

However, it is challenging to detect novel Coronavirus (nCov) infections at an early stage with the help of X-ray and CT scan images using deep learning. However, at a later stage, the task of radiologists in screening COVID-19 patients can be eased. Deep learning as an emerging concept is gaining popularity in the field of medical imaging. Before discussing more details about the deep learning paradigm, let us find out the relationship between neural network (NN), deep learning (DL), Machine Learning (ML), and Artificial Intelligence (AI) as shown in Figure 2.

Mei et al. [4] presented an AI-based solution for minimizing the RT-PCR method's time. They have integrated chest CT finding with several other factors, namely, symptoms and laboratory testing for rapid diagnosis of COVID-19. The system was claimed to be a more powerful tool for radiologists if CT images and clinical history were available. The reason behind the integration of other parameters with CT findings is to provide higher accuracy because CT findings alone are not enough to predict the infection. In some cases, early CT findings can be standard for an infected person, so, to minimize the risk of spreading the disease, it is foremost required to integrate some other parameters to have a clear idea.

The authors first developed a convolutional neural network (CNN) model to learn the characteristics of CT images. The process is put into action by the classification of COVID-19 patients using three different classification techniques, namely, Support Vector Machine (SVM), Multilayer Perceptron (MLP), and Random Forest. The performance of MLP was better than those of the other techniques under consideration.

Fong et al. [5] developed a model using Composite Monte Carlo (CMC) for making decisions under the high uncertainty of 2019-nCov. We know that, in the pandemic of COVID-19, every Government is supposed to make crucial decisions to save its citizens' essential lives, but, due to the uncertain behavior of 2019-nCov, it seems a challenging task. CMC can forecast by combining data from small data sources, followed by drawing probability distributions. The authors have significantly used this property of CMC, followed by enhancements using DL and fuzzy rule induction. MC is suitable to model epidemics such as COVID-19 because their data are generally changing over time. MC provides output in terms of probability distributions of expected outcomes. The work of Fong et al. [5] is based on the Group of Optimized and Multisource Selection (GROOMS), which is applied to select a Machine Learning model based on accuracy. They have analyzed the data collected from the Chinese Center for Disease Control and Prevention^1^(CCDC). Their parameters of interest were only a few, namely, the number of people affected by and cured of COVID-19. However, these parameters' values depend on various other parameters, namely, social factors and psychological factors. The method was followed by fuzzy rule induction (FRI), which further investigates the logic behind the epidemic. Their goal was to estimate the cost needed for controlling and planning during these epidemics. Experimental results have shown that the novel methodology can forecast the direct cost requirements for dealing with COVID-19 epidemics. On the other hand, Peng and Nagata [6] analyzed the trend of COVID-19 pandemic data of the twelve most affected countries for predicting the number of COVID-19 cases using Machine-Learning-based approaches. They have emphasized the need for utmost caution while applying Machine Learning models in decision making, especially during the COVID-19 pandemic. On the other hand, Mehta and Shukla [7] presented a pandemic analysis using AI and big data analytics.

### 2.1. Some AI-Enabled Tools for Coping with a COVID-19 Outbreak

AI-enabled tools are getting popular in the healthcare domain due to their tremendous applications. Many companies are running their businesses in the healthcare sector by providing solutions to common problems using AI. Current applications of AI, namely, radiology and diagnosis, are so specific that they may not be suitable to predict a global pandemic like COVID-19. However, few companies like BlueDot [8] and Metabiota [9] claimed that their AI-enabled solutions can identify, quantify, and mitigate the risks due to the COVID-19 outbreak.

#### 2.1.1. BlueDot

The AI-enabled tool of BlueDot [8] can perform predictions on outbreaks of infectious diseases. It collects data from numerous sources using AI and Natural Language Processing (NLP) capabilities. As per its website, BlueDot was the first to intimate its client about COVID-19 risk via their “insights” platform. Its Big Data processing capabilities collect data from more than 10,000 sources over 60 languages every day [10]. Primary sources include air travel data, population density, national statistics reports, World Factbook, global infectious disease alert, climate data, and animals' disease reservoirs. After collecting data from such heterogeneous sources, this AI-enabled start-up company processes this data by applying some preprocessing and clustering techniques for identifying patterns of interest, namely, outliers and hotspots. This data is further employed to train their powerful system for sending notifications to their customers.

#### 2.1.2. Metabiota

Metabiota [9] works by integrating several technologies like AI, NLP, and Big Data to make predictions regarding disease outbreaks. It works by collecting data from several sources, analyzing them using advanced analytical tools, and making predictions about outbreaks. It also searches data from social media platforms to observe human behavior due to COVID-19 pandemic [10]. This kind of behavior analysis is then supplied to their prominent clients (i.e., insurance companies) so that they can identify potential customers for investing in insurance products.

#### 2.1.3. Chatbots

Chatbots can also play a critical role in screening patients before sample collection. Due to the COVID-19 pandemic, pathological laboratories (identified as COVID-19 test/sample collection center) face a huge crowd. To minimize this crowd, these labs are filtering patients by first putting them under NLP-enabled chatbot to answer a few essential queries; and one can decide the severity or urgency of being tested. Their chatbots are so powerful in analyzing the responses of patients in real time and suggesting the preliminary diagnosis. Patients on their own can take advantage of these chatbots at their home before proceeding to hospitals/laboratories.

#### 2.1.4. Qure.ai

Qure.ai [11], a US-based company, is offering several solutions in the field of healthcare. To cope with the pandemic of COVID-19 using AI, they have devised two special tools, namely, “qXR” and “qScout-EMR.” “qXR” tool is meant for COVID-19 progression monitoring. This automated tool monitors the progression of infected patients daily. It automatically estimates the affected lung area and tracks changes. “qScout-EMR,” on the other hand, is providing a pandemic response care platform. All registrations of infected persons are done using this tool and are accessible via any mobile or laptop. The registration step adds all linked contacts that can be at risk. It monitors their health by daily symptom checking and sending intimations to all concerned automatically.

#### 2.1.5. AlphaFold

DeepMind [12], founded in 2010 and further acquired by Google in 2014, is a famous AI-enabled company working for advancing the state of the art. DeepMind's “AlphaFold” is an AI-enabled protein structure prediction system, shown in Figure 3. The core of AlphaFold is its CNN model trained with genomic data extracted from Protein Data Bank (PDB). It works by finding out the distributions among several pairs of residues in a protein because disease predictions rely heavily on protein structure. The distribution calculation is antecedent to the estimation of the proposed structure.

#### 2.1.6. RADLogics

RADLogics [13] has presented its AI-based CT image analysis tools for accurate and automatic identification of COVID-19. Their AI-based analysis also suggests a corona score for measuring a patient's progression and recovery time. Another AI-based solution called “Virtual Resident” can analyze X-ray, CT scan, MRI, and ultrasound scans. Some researchers [13] also deployed a deep-learning-based model for COVID-19 classification from CT scan images using pretrained AI systems of RADLogics as their subsystem.

#### 2.1.7. Aarogya Setu

To help reduce the spread of COVID-19 in India, the Government of India (GOI) launched the Aarogya Setu mobile app [14] on April 02, 2020. Aarogya Setu app provides many facilities based on Bluetooth and GPS, such as contact tracing of COVID-19 patients, hotspot mapping, and providing other important information relevant to COVID-19. Over 215 million users were taking benefits from this app as of April 05, 2022. After installation, the user must complete a self-assessment test by answering some simple questions on symptoms of cough, fever, difficulty in breathing, hypertension, heart disease, diabetes, lung disease, travel history, interaction with any COVID-19 patient, and so forth. Based on users' answers, this app collects location-related data via Bluetooth and GPS so that the Government can track the patient and notify other users within that region. Along with COVID-19 tracking, the app provides several other facilities to the citizens, that is, e-pass (permission for traveling to other states and districts during lockdown period) generation, COVID-19 updates, COVID-19 helpline, useful resources, list of laboratories approved by GOI for COVID-19 testing, essential links for donations to PM care fund, and notifications related to COVID-19 patients within the radius of 500 m to 10 km. The app is available to be used in twelve languages of India, and its code was also released to be open source by GOI on May 26, 2020.

#### 2.1.8. AI4COVID-19

Imran et al. [15] developed an AI-engine-based app to distinguish between a regular cough and a COVID-19 cough by analyzing cough samples. Cough is a common symptom of suffering from cold, and that is why cough alone cannot be the key-decisive parameter to identify that a person is suffering from COVID, but it can help patients perform initial screening on their own in just a few moments. During the COVID-19 pandemic, such apps present themselves as the best usage of technologies.

As per the availability of progressive cough data, the accuracy of this app may improve. The app is also not clinically approved but is based on features of distinct respiratory syndromes of cough. The app works by collecting cough samples that are input for the pretrained AI engine to recognize the type of cough based on features. The overall architecture of AI4COVID-19 is depicted in Figure 4. Initially recorded cough samples are converted to Mel-spectrogram using Cepstral analysis. The result of this phase is the input images for the CNN model for cough detection. Experimental detail shows 90% accuracy of the AI4COVID-19 app for the identification of COVID and non-COVID cough. Several other applications which are applied by many countries for tracing COVID-19 are summarized by Lalmuanawma et al. [16].

## 3. Deep-Learning-Based Identification of COVID-19 and Pneumonia from CT Scan Images

Detecting COVID-19 from images alone is a challenging task. Due to the sudden outbreak of COVID-19, radiologists and hospitals are feeling overburdened. This type of burden on the healthcare sector is correlated directly with COVID-19 mortalities [17]. On the other hand, deep learning methodologies are trying to reduce this burden by screening COVID-19 patients at an early stage. In a short period, plenty of researchers have developed CNN models for faster and reliable patients' screening to minimize the time required for disease identification. CT scan analysis is one of the predominant investigations for the screening of COVID-19 patients. The importance of CT scan images is observed easily from several clinical case study reports. Lin et al. [18] discussed the importance of CT scan images in identifying asymptomatic patients of Novel Coronavirus Pneumonia (NCP). The reported patients were asymptomatic with no preexisting diseases. However, multiple ground-glass opacities (GGO) were located with the help of High-Resolution CT (HRCT). One of the patients was 61 years old, and that patient remained without any complications and had no symptoms, namely, fever, fatigue, cough, myalgias, headache, tiredness, sputum production, hemoptysis, or diarrhea. The patient also had no history of smoking and no history of other diseases, namely, cardiovascular disease, diabetes, and hypertension. The patient was treated with oral antiviral drugs only. Fortunately, after the 23rd day of admission, the patient's bilateral pulmonary lesions and pleural effusions got resolved.

DL-based implementation is used for preparing detailed clinical reports of patients as well. In this regard, Cao et al. [19] presented detailed illustrations of two COVID-19 positive patients using voxel-level DL-based segmentation of CT scan images based on U-Net [20]. Keeping in mind the importance of CT scan images, this section highlights some of the works that focused on identifying COVID-19 and pneumonia from chest CT scan images using deep-learning-based paradigms. Although CNNs provide several metrics by which one can analyze their performances, the work discussed in this paper is mainly focused on analyzing classification metrics. One of the prime metrics to measure the classification performance is the confusion matrix, shown in Figure 5.

The confusion matrix summarizes correct versus incorrect predictions of a classification model, where predicted observations are matched with the actual ones. TP, FP, FN, and TN are explained as follows:

- True Positive (TP): positive prediction of positive observation.
- False Positive (FP): positive prediction of negative observation.
- False Negative (FN): negative prediction of positive observation.
- True Negative (TN): negative prediction of negative observation.

These metrics are further utilized to provide the classification performance in terms of precision, specificity, sensitivity, accuracy, and so forth described as given in the five following equations:

(1) $$\begin{array}{c} \text{precision}=\frac{\text{TP}}{\left(\text{TP}+\text{FP}\right)}\text{,} \end{array}$$

(2) $$\begin{array}{c} \text{Sensitivity}=\frac{\text{TN}}{\left(\text{TN}+\text{FP}\right)}\text{,} \end{array}$$

(3) $$\begin{array}{c} \text{Specificity or Recall}=\frac{\text{TP}}{\left(\text{TP}+\text{FN}\right)}\text{,} \end{array}$$

(4) $$\begin{array}{c} \text{Accuracy}=\frac{\left(\text{TP}+\text{TN}\right)}{\left(\text{TP}+\text{TN}+\text{FP}+\text{FN}\right)}\text{,} \end{array}$$

(5) $$\begin{array}{c} F1\text{Score}=\frac{2\times \text{precision}\times \text{Recall}}{\left(\text{Precision}+\text{Recall}\right)}\text{.} \end{array}$$

In this paper, the authors presented a comparison based on classification accuracy of several deep learning models for classifying CT scan as well as X-ray images to COVID-19 and non-COVID-19 images.

Wang et al. [21] deployed an AI-based system that is capable of automatically detecting COVID-19 from CT scan images. Their system has achieved a sensitivity of 0.98 and is installed in 16 hospitals, screening 1300 cases per day. The system is doing two main intended tasks, namely, reducing healthcare burden during screening and fulfilling the lack of experienced radiologists. Based on their earlier developed deep learning models, they have selected the best model for this task. The data of COVID-19 patients were taken from 5 hospitals in Wuhan and Beijing. After collecting relevant data, annotations for lesions (if any) were processed, followed by several preprocessing techniques (normalization, window width, window width adjustments, lung segmentation, etc.). The deep learning architecture of their system is mainly divided into two models, namely, segmentation and classification. The segmentation model is used for obtaining lung regions, and the classification model determines COVID-19 positivity in these regions. For both segmentation and classification models, they have selected the best models out of their previously developed models. The combined 3D U-Net++ [22] (segmentation model) and ResNet50 [23] (classification model) achieved best area under the curve (AUC) of 0.991.

Zheng et al. [24] developed a novel CNN model called DeCoVNet for detecting COVID-19 from chest CT images. The model first segments the CT images using a pretrained U-Net [20], and then these segmented images are fed into the DL model for COVID-19 prediction. Along with segmented images, they have considered several other factors, namely, clinical signs, travel and disease history, and laboratory examinations. The ground truth label was applied as per the decision made by expert radiologists. The input to DeCoVNet is CT volume and its corresponding lung mask (generated by U-Net [20]). 3D lung mask contributes toward reducing background information to achieve higher accuracy. Original CT volume is combined with the 3D lung mass volume to make a final volume followed by resampling into a 224 × 336 resolution. Due to limited data availability, data augmentation has been applied. These resampled images serve as input for training the network. DeCoVNet consists of three main parts, namely, network stem, 3D residual blocks (ResBlocks), and a progressive classifier (ProClf). The network stem consists of 3D convolution using a kernel of a 5 × 7 × 7 size and batch norm and pooling layers. Meanwhile, in the second step, from each ResBlock, a 3D feature map is being passed into 3D convolution. Finally, ProClf performs the classification of images using three 3D convolution layers and a fully connected layer with a softmax activation function. The overall pipeline of DeCoVNet is shown in Figure 6. For validating the experimental study, images of 630 CT scans were considered. Out of 630 CT scans, 499 were used for training and the rest for testing. The results of the experimental study are promising, which in turn may contribute to the healthcare sector.

Song et al. [25] proposed a deep learning model for the identification of COVID-19 from chest CT scan images. They first collected CT scan images of 88 COVID-19 patients, followed by preprocessing filling blank regions in the lung images. Top-k detail from CT scan images was extracted using Details Relation Extraction Neural Network (DRE-Net) and then final prediction was performed using aggregation. However, the model was able to achieve the classification accuracy of only 86%.

Zhang et al. [26] constructed a novel deep-learning-based model for the rapid diagnosis of COVID-19 from an extensive CT image database of 3,777 patients. The overall work is comprised of two main models, namely, lung segmentation and analysis. In lung-lesion segmentation, the lung lesions are segmented from the background using DeepLabv3 to create a lung-lesion map. The lung-lesion map is further utilized for the classification of CT segments and achieved an overall classification accuracy of 92.49%.

Pretrained models are playing a pivotal role in deploying models for COVID-19 identification. Kini et al. [27] employed the concept of transfer learning by proposing an ensemble deep learning model and achieved an overall accuracy of 98.98%. Li et al. [28] developed a deep learning model called COVNet (based on ResNet50 [23]) for detecting COVID-19 by extracting features from 4356 3D chest CT examinations (collected from 6 hospitals). Out of these images, 30% were of COVID-19-positive patients (confirmation by RT-PCR), 40% of community-acquired pneumonia (CAP), and the rest 30% of nonpneumonia. They have used the 3D CT scan slices as input for training the model and developed a feature map from features extracted from these slices. The feature extraction phase is then followed by a max-pooling operation for combining features of these slices. Finally, a fully connected layer generates a feature map followed by the generation of probability score by a softmax activation function. Their model was able to present the specificity of 96% and AUC of 0.96 for COVID-19 identification.

Ardakani et al. [29] presented a study of ten CNN models for classification of COVID-19 from other types of pneumonia from CT scan images. Out of ten well-known CNN models, the performances of ResNet-101 [23] and Xception [30] were found to be better compared to the others. ResNet-101 achieved 99.51% accuracy, whereas Xception achieved 99.02% in classifying COVID-19 cases from non-COVID-19 cases. They have also analyzed radiologists' performance for the same purpose and reported moderate performance with a classification accuracy of 83.33%. It is evident that not only are computational models, especially deep learning models, able to save a significant amount of time in reading the radiographical images but also they provide accurate results.

Xu et al. [31] presented an automated deep learning model (based on ResNet18) for COVID-19 classification from 3D CT scan images. The experimental evaluation was done on 618 CT samples, out of which 219 images were of 110 COVID-19 patients, 224 of influenza patients, and 175 of healthy personnel. These 3D CT images were then segmented for identification of required region of interest. Feature extraction was done from segmented images using ResNet18, followed by pooling operation for dimension reduction and to prevent overfitting. The output is then converted to a feature vector followed by a fully connected layer that provides the final classification of images into three classes: COVID-19, influenza, and healthy. The model was able to achieve an overall classification accuracy of 86.7% only.

Chen et al. [32] presented a deep learning model (based on U-Net++ [22]) for COVID-19 classification from High-Resolution CT (HRCT) scan images. A dataset of 46096 CT images of 106 patients was used for evaluating the performance of the model. Three experienced radiologists did the labeling on infected regions. The model has achieved the per-patient classification accuracy of 95.24% and per-image classification accuracy of 98.85%. However, some inconsistencies were observed between the evaluations performed by a radiologist and their model.

Shan et al. [33] developed a 3D convolutional neural network called VB-Net (based on V-Net [34]) for COVID-19 classification from CT scan images. As compared to V-Net, VB-Net has shown more efficiency. VB-Net consists of two phases, namely, downsampling and feature extraction and upsampling and feature integration. A total of 549 CT images were considered for the study, out of which 300 were used for testing and 259 for training. Testing and training contained a significant number of lung infections and they were collected from different CT scan centers. Based on segmentation results by VB-Net, the study follows a statistical analysis of the percentage of infection (POI) in lung and bronchopulmonary segments. Comparative analysis between automatic segmentation and manual segmentation yields a mean POI estimation error of 0.3%.

Huang et al. [35] presented a deep learning model (based on U-Net [20]) for the classification of chest CT scan images. Generally, deep learning models only prove the necessary information about whether a patient is affected by a disease. However, their model classified CT images into four categories (i.e., mild, moderate, severe, and critical) with the help of evaluation performed by both automatic segmentation and radiologists. A chest CT scan of 842 COVID-19 confirmed patients was considered in the experimental evaluation. For feature extraction, U-Net [20] uses downsampling for reducing the 512 × 512 image to a 16 × 16 × 256 feature map and upsampling to 512 × 512 × 2 for lesion localization.

Wang et al. [36] presented a deep learning algorithm by fine-tuning the pretrained Inception model to classify chest CT images. They have used 1,065 images for the experimental study, out of which 325 images were of pathogen-confirmed COVID-19 patients. Their algorithm consists of three main components, namely, image preprocessing, feature extraction, and classification. Overall, network architecture can be viewed as a two-phase network model, where the first phase is responsible for generating a one-dimensional feature vector, and later a fully connected network performs the final classification. The overall classification accuracy (89.5%) of their model is further compared with the predictions made by two skilled radiologists. The performance of thier model was found to be better than the performance of radiologists. Pan and Guan [38] also summarized some expected changes in the patients using CT scan images. CT manifestations can represent several features (lung GGOs, pulmonary consolidation, nodules, etc.) that can help detect 2019-nCov. Pathak et al. [37] presented a deep-transfer-learning-based model using ResNet50 [23] for detecting COVID-19 cased from CT images. Their model was able to achieve a test accuracy of 93% only. Meanwhile Wu et al. [39] presented a deep-learning-based multiview fusion model capable of analyzing age-based subgroups of COVID-19 cases from CT images. The summary of several deep-learning-based models used for diagnosis of COVID-19 from CT scan images is presented in Table 1 along with their classification accuracies. However, the datasets used in these works may not be the same.

## 4. Deep-Learning-Based Identification of COVID-19 and Pneumonia from X-Ray Images

Chest X-ray images also have the capabilities to show the symptoms of lung infections. However, as compared to CT images, X-ray images are less sensitive [40]. In most cases, the chest X-rays are reported to be normal during the disease's initial stages [41]. At later stages, some abnormalities in terms of diffuse and peripheral lung involvements have been observed. Nowadays, plenty of research is considering X-ray images to determine whether a person is suffering from COVID-19 or not. In this section, the authors tried to cover some of the works related to COVID-19 and pneumonia identification from chest X-ray images using deep-learning-based paradigms.

Aftab et al. [42] proposed an LSTM-based model to classify chest X-ray images into three classes, namely, normal, influenza, and COVID-19. With the incorporation of LSTM, their model was able to achieve 98% accuracy. Another LSTM-based model to detect COVID-19 from hybrid images was proposed by Irfan et al. [43]. Their hybrid deep neural network (HDNN) was equipped with a CNN for automated feature extraction and an LSTM for dealing with vanishing gradients. The HDNN was able to provide 99% classification accuracy on hybrid images. Almalki et al. [44] presented a novel deep-learning-based method called CoVIRNet (COVID Inception-ResNet model) for COVID-19 identification from X-ray images. The proposed model was able to achieve a classification accuracy of 97.29% using the Random Forest classifier. Zhang et al. [45] developed a new reliable deep learning model for fast screening of COVID-19 patients. The model works by detecting anomalies from chest X-ray images with 96% accuracy for symptomatic patients and 70.65% for asymptomatic persons. Their model consists of three main phases, namely, backbone network, classification, and anomaly detection. The purpose of the backbone network is to extract useful features from X-ray images. These features act as inputs for classification and anomaly detection. The results presented by them are promising, with a limitation of a 30% false positive rate. Deep learning has many applications in the healthcare sector. Panwar et al. [46] also presented a deep-learning-based model called nCOVnet for detecting COVID-19 from X-ray images. Their model is based on the concept of transfer learning where they have used top layers of VGG16 [47] and later customized with other layers. Experimental analysis on 337 X-ray images (192 COVID-19-positive images) presented a classification accuracy of 97.62%.

Stephen et al. [48] have also presented an efficient approach for pneumonia classification using deep learning. Their dataset contains 5,856 anterior-posterior chest X-ray images of pneumonia patients aged 1 to 5 years. To make the dataset adequate and reduce the chances of overfitting, several augmentation techniques were employed. Their model contains two main parts, namely, feature extractor and classifier. Feature extractor contains four convolution layers (conv3 × 3, 32; conv3 × 3, 64; conv3 × 3, 128; and conv3 × 3, 128), max-pooling layer of a 2 × 2 size, and ReLU activation function. For classification, the dense layer uses the 1D feature vector as provided by the flattening process. Experimental results showed that their model could classify pneumonia and nonpneumonia images with a training accuracy of 0.95 and validation accuracy of 0.93. Wang and Wong [49] developed a novel deep learning model called COVID-Net for the detection of COVID-19 from chest X-ray images. They have classified chest X-ray images into four classes, namely, normal, bacterial infection, non-COVID viral infection, and COVID infection. The architecture design is mainly based on the projection-expansion-projection pattern. Despite adequate dataset consisting of 5941 chest images of 2839 patients collected from two growing public datasets, they achieved only 83.5% test accuracy.

DeTraC, a new method for detection of COVID-19 from chest X-ray images, has been presented by Abbas et al. [50]. DeTraC uses a threefold approach consisting of pretrained CNN models for feature extraction followed by class decomposition, training using gradient descent optimization, and classification. Experimental results on X-ray images showed a classification accuracy of 93.1% using VGG19 [47].

Zebin and Rezvy [51] used several pretrained CNNs for extracting features from chest X-ray (CXR) images and achieved 96.8% accuracy using EfficientNetB0 for COVID-19 classification. Apostolopoulos et al. [52] also presented the classification of COVID-19 disease using state-of-the-art MobileNetV2 [53] on 3905 CXR images. Training the CNN from scratch can also lead to higher accuracy as depicted in their experimental results for classification of COVID and non-COVID cases. Along with COVID, their dataset consists of images of five other diseases and normal CXR images. Concerning the 2-class classification problem, their model gained an overall accuracy of 99.18% compared to 7-class accuracy of 87.66%.

Instead of developing deep learning models from scratch, pretrained models are also gaining popularity. In this regard, Toğaçar et al. [54] presented a model based on MobileNetV2 [53] and SqueezeNet [55] followed by SVM-based classification for classifying COVID-19-affected chest X-ray images from normal and pneumonia images.

The deep learning model MobileNet is designed to perform object detection and classification for low hardware devices. MobileNet uses the ReLU activation function for providing nonlinear outputs. SqueezeNet [55], on the other hand, provides faster results by reducing the number of parameters, which leads to a reduction in overall model size. It contains a cascade of convolution, pooling, and fire layers. They have applied the concept of image reconstruction using the fuzzy color technique to remove noise. The images produced by the fuzzy color technique are further mixed with original images for the creation of a new dataset. 1000 features were generated with both MobileNet and SqueezeNet on the new dataset, followed by efficient features using Social Mimic Optimization (SMO). The overall pipeline of their work is depicted in Figure 7.

Experimental analysis on the 70 : 30 ratio of training and testing dataset claimed 99.27% accuracy using both models. Ozturk et al. [56] proposed a deep learning model based on the YOLO pretrained model called DarkCovidNet to automatically identify COVID-19 cases from X-ray images with an accuracy of 98.08% for binary classes (COVID and non-COVID). However, one of the essential requirements for a deep learning model (large dataset) is still missing. They have used a database consisting of 127 X-ray images of COVID-19-positive patients . Also, most of the patients' age information is unknown, and the age was approximated to be 55 in their experimental evaluation. However, 1000 images from another dataset named ChestX-ray8 are also considered in the study, but they all do not belong to COVID-19 patients. Their model contains 17 convolutional layers, followed by BatchNorm and LeakyReLU operations. For updating weights, the Adam optimizer is being used along with the cross-entropy loss function. Their experimental results are based on an 80 : 20 ratio of training versus testing data using 5-fold cross-validation and 100 epochs. After classifying images into COVID-19 and no findings, they have used HeatMap to identify the lesions, and the same was presented before expert radiologists for final verification, as shown in Figure 8. This final step provides strength to validate the proposed model.

Ghosal and Tucker [57] presented a Bayesian deep learning classifier that uses pretrained ResNet50V2 to classify COVID-19 images from 5941 chest X-ray images. Their objective was to help radiologists estimate the uncertainty of deep learning models for reliable prediction of diseases. Especially for a beginner radiologist, deep learning models can contribute to increasing overall prediction accuracy.

On the other hand, Narin et al. [58] presented a deep learning model for the identification of COVID-19 using three existing deep learning models, namely, ResNet50 [23], InceptionV3 [59], and InceptionResNetV2 [60], from X-ray images as shown in Figure 9.

Their models need no separate feature extraction; instead, they use the transfer learning capabilities that provide adequate accuracy even in fewer data. Their experimental analysis depicted higher classification accuracy of 98% using ResNet50 [23] compared to 97% and 87% accuracy using InceptionV3 and InceptionResNetV2, respectively.

Sethy et al. [61] also presented a framework for the identification of COVID-19 from chest X-ray images. Their model extracted features from thirteen existing CNN models followed by SVM classification. The classification problem presented here is a three-class problem intended to classify chest X-ray images into three classes, namely, healthy, pneumonia, and COVID. A total of 381 X-ray images (127 of each category) have been considered in the experimental study. RestNet50 [23] model was able to present maximum classification accuracy as compared to other models under consideration.

Hemdan et al. [62] presented a framework that takes advantage of the existing seven deep learning models, namely, VGG19, DenseNet201 [63], MobileNetV2, Xception, ResNetV2, InceptionResNetV2, and InceptionV3. They have considered chest X-ray images of 50 patients only, out of which 25 patients were COVID-19-positive. Experimental results show higher accuracy of 90% in the cases of VGG19 and DenseNet201.

Khan et al. [64] also presented a deep learning model called CoroNet based on a pretrained Xception model for the classification of chest X-ray images. Xception is pretrained on the ImageNet dataset and consists of 71 deep layers connected in a residual manner, which avoids vanishing gradients. Their work is classified into three main scenarios, namely, four-class, three-class, and two-class classification. Their experimental analysis on public datasets [2] revealed an overall classification accuracy of 89.6%.

Rahimzadeh and Attar [65] trained various CNN models and presented a concatenated network using Xception and ResNet50V2 for classifying X-ray images into three classes, namely, COVID-19, pneumonia, and normal. Xception contains several inception layers which are formed from depthwise convolution followed by a pointwise convolution operation. ResNet50V2, on the other hand, is a modified version of ResNet50 [23], whose performance is better than that of ResNet50. Their input dataset consists of 180 images (300 × 300 pixels) of COVID-19-positive patients. Both Xception and ResNet50V2 produced an equal-sized 10 × 10 × 2048 feature map from their feature extractors. These feature maps are then concatenated, followed by a convolution layer. Confusion matrices showed that the concatenated network achieved 99.50% accuracy in classifying COVID-19 images with an overall accuracy of 91.4%.

Chowdhury et al. [66] presented a comparative study of various deep learning models, namely, DenseNet201, ResNet18, SqueezeNet, MobileNetV2, InceptionV3, ResNet101, CheXNet [67], and VGG19, for classifying chest X-ray images into three different classes, that is, normal, COVID-19, and viral pneumonia. They have created a COVID-19 dataset of chest X-ray images. For doing this, they have received “Winner of COVID-19 Dataset Award” by Kaggle. Testing and training accuracies of four different CNN models have been presented. SqueezeNet achieved higher testing accuracy of 98.3%, whereas ResNet18 achieved higher training accuracy of 99.5%. Apostolopoulos et al. [68] incorporated the concept of transfer learning and evaluated five well-known CNN models (VGG19, MobileNetV2, InceptionResNetV2, Inception, and Xception) on two chest X-ray databases for classification of COVID-19. VGG19 and MobileNetV2 were able to achieve higher accuracy of 98.75% and 97.40%, respectively, compared to other models in the case of two-class classification. For the three-class classification task, VGG19 achieved the highest accuracy of 93.48% among all other models under study.

Altan and Karasu [69] developed a hybrid model called EfficientNetB0 using deep learning, 2D curvelet transformation, and Chaotic Salp Swarm Algorithm (CSSA) for screening COVID-19 cases from X-ray images. Experimental results on X-ray images of 219 COVID-19 patients showed that the hybrid model has achieved the classification accuracy of 99.69%. At the same time, Brunese et al. [70] presented a transfer-learning-based model for classifying COVID-19 images from X-ray images with an accuracy of 97%. Ucar and Korkmaz [71] also presented a deep learning model based on light pretrained SqueezeNet for classifying COVID-19 from X-ray images. Their system firstly augments the raw dataset in an offline manner, followed by training of deep-SqueezeNet that takes advantage of Bayesian optimization and then tests the network for final decision making. The main reason behind using Bayesian optimization is to optimize hyperparameters automatically. The Bayesian optimization task calculates the posterior probability *P*(*D|L*) of a deep learning model using learned data. Experimental results on the COVIDx public dataset showed 100% classification accuracy in COVID X-ray images with an overall classification accuracy of 98.26%. Mahmud et al. [72] proposed a deep-learning-based model called CovXNet to extract various features from chest X-ray images. They first trained their model with chest X-ray images of traditional pneumonia followed by COVID-19-caused pneumonia because they possess almost the same kind of imaging features. Experimental results have shown that their system can provide multidilation classification with an accuracy of 97.4%.

On the other hand, Pereira et al. [73] also presented a deep learning model based on InceptionV3 for the identification of COVID-19 from chest X-ray images. They have performed multiclass classification using five famous classifiers and achieved an *F*1-score of 0.89 in classifying COVID-19 from another type of pneumonia. Performance analysis of several deep learning models for classification of COVID-19 from X-ray images is presented in Table 2. However, the datasets used in these works may not be the same. During this pandemic, plenty of researchers came with several pretrained and transfer-learning-based approaches for the classification of COVID-19 from chest X-ray and CT samples [74–78].

Along with CT and X-ray-based examinations, some clinical observations also play an essential role in detecting diseases. In this regard, Hosseiny et al. [67] presented a comparative study of clinical and radiological features of COVID-19 with existing SARS and MERS diseases. They highlighted the importance of early CT findings for the diagnosis of COVID-19. Li et al. [79] presented an analysis of both clinical manifestations and COVID-19 imaging. On the other hand, Shah et al. [80] presented a comprehensive survey of several computational approaches for detection of COVID-19 from medical images.

## 5. Other Computational Approachesfor COVID-19

Plenty of AI-based, statistical, and technological solutions are also provided by researchers in the area of COVID-19 research. Digital technology has several applications that can help plan and respond to COVID-19 pandemic [68]. This section highlights some of the works related to computational models for diagnosing and predicting COVID-19.

### 5.1. Machine-Learning-Based Approaches

Machine Learning approaches learn by extracting useful features from the data and can predict the futuristic trends/patterns using that learning. These approaches proved themselves in providing support to the clinical diagnosis.

To assist the quick diagnosis of COVID-19 and analyze the epidemic trends, several Machine-Learning-based solutions have been presented by researchers. For a quick and accurate diagnosis of COVID-19, a Random Forest (RF) based tool has been developed by Wu et al. [81]. The tool has extracted 11 blood indices from clinical blood test data and proved its validity by achieving 96% accuracy. Shi et al. [82] also developed a Random Forest based approach for automatic classification of CT samples based on infected lesions' size. Adjuik et al. [83] presented a Machine Learning approach based on neural network to generate protein vectors for preventing COVID-19.

On the other hand, Qi et al. [84] developed a model using Random Forest and linear regression for predicting the approximate stay of patients in the hospital due to COVID-19. Another Random Forest based approach for identifying significant predictors and subsequent risk factors on mortality has been presented by Sarkar and Chakrabarti in [85]. They have analyzed the clinical data of COVID-19 patients and presented that age is one of the essential parameters responsible for mortalities.

Support Vector Machine (SVM) is a famous classification approach that can assist in clinical diagnosis in early detection of COVID-19. Batista et al. [86] performed a comparative study of five Machine-Learning-based approaches, namely, ANN, RF, SVM, Logistic Regression, and Gradient Boosted Trees. They have analyzed the clinical observations of 235 patients and presented all five algorithms' predictive accuracy under consideration. Among these approaches, SVM was able to predict the positivity of COVID-19.

On the other hand, Singh et al. [87] analyzed the daily confirmed cases data of the five most affected countries and presented one-month predictions using Autoregressive Integrated Moving Average (ARIMA) and Least Square Support Vector Machine (LS-SVM) approaches. Experimental results have shown the higher performance of LS-SVM by predicting a rapid rise in COVID-19 cases. Machine Learning approaches can be applied to viral sequence datasets for obtaining useful information. In this regard, Bzhalava et al. [88] used Artificial Neural Network (ANN) and Random Forest techniques for classifying viral and nonviral sequences from metagenomic datasets. Ardabili et al. [89] presented a study of Machine Learning and soft-computing-based approaches for predicting COVID-19. They observed that Multilayer Perceptron and Adaptive Network-Based Fuzzy Inference System (ANFIS) provided the best classification accuracy for predicting COVID-19. Hasan et al. [90] utilized Q-Q plot and ARIMA model to present the death rate based on time-series data of different states of India. Many other researchers [91–99] have presented the applications of Machine Learning approaches for early diagnosis and predicting the trends of COVID-19. Wang et al. [100] presented the epidemic trend using logistic and time-series prediction model called FbProphet. They have analyzed the country-level daily COVID-19 data from John Hopkins University. The “Prophet” is a Facebook forecasting model that predicts the epidemic trends based on trend function, periodic term, influence, and the error term. First, they integrated the most recent data into the logistic model and then fed the cap values into the Prophet model to generate epidemic curves. Tuli et al. [101] emphasized the applications of Machine Learning and cloud-computing-based approaches in predicting the trend and the growth of COVID-19 from country-wise data obtained from Our World in Data [102]. They have applied five different distributions on that data and observed that the Inverse Weibull function provides the best fitting distribution using the iterative weighting approach. There are numerous applications of AI in the COVID-19 pandemic. In this regard, Vaishya et al. [103] presented several applications of AI for coping with the COVID-19 pandemic. The main applications highlighted by them include early diagnosis, treatment monitoring, contact tracing, cases/mortality projection, drug development, reducing the workload of health workers, and prevention of disease. Kumar et al. [97] analyzed several key parameters responsible for COVID-19 outbreak using two famous Machine Learning algorithms, namely, multiple regression analysis and multilayer feedforward neural network. They have analyzed several parameters for finding out correlation with two main parameters, that is, total mortalities and total cases. Meraihi et al. [104] presented a critical analysis of several Machine-Learning-based approaches for detection, diagnosis, and prediction of COVID-19. To discover the COVID-19 patterns from recovered patients, a case study of Saudi Arabia was presented by Alafif et al. [105] using Association Rule Apriori (ARA) algorithm.

### 5.2. Industry 4.0 Based Approaches

The fourth industrial revolution, termed as Industry 4.0, also has the potential to provide solutions to some problems during the COVID-19 pandemic. In this regard, Javaid et al. [106] reviewed several technologies of Industry 4.0 and explored their applications in minimizing the effects of the COVID-19 outbreak. They have presented the applications of 10 leading technologies of Industry 4.0, namely, AI, IoT, Big Data, cloud computing, Virtual Reality, Holography, autonomous robotics, 3D printing, 3D scanning, and Biosensors, effectively. One of the essential aspects of Industry 4.0 is Big Data, which provides a massive amount of healthcare records, bringing the insight/surveillance of pandemics like COVID-19 [107]. The supply chain sector is one of the critical sectors which was critically affected during the COVID-19 pandemic. Potentials of Industry 4.0 can minimize the impact of several challenges on the supply chain sector [108, 109]. Nowadays, the integration of IoT in medical technologies enables easy and transparent monitoring of patient's health [110]. Nowadays, this integration is sometimes referred to as the Internet of Medical Things (IoMT). Swayamsiddha and Mohanty [111] analyzed several applications of Cognitive Radio on IoMT. Modern technologies have several applications in pandemics, namely, disease tracking, health monitoring, predicting protein structures, drug discovery, and social awareness. Kumar et al. [112] and Chamola et al. [113] presented a comprehensive review of such technologies for dealing with the COVID-19 pandemic. On the other hand, Devi et al. [114] presented several applications of flying ad hoc networks (FANET) during COVID-19 pandemic.

### 5.3. Statistical Approaches

As compared to AI-based approaches, statistical techniques can provide detailed insights of daily, cumulative, country-wise data of COVID-19. Plenty of research has been carried out by researchers using statistical techniques to analyze the COVID-19 daily confirmed data. Zhang et al. [115] presented automated detection of COVID-19 using the “AI Intelligent Assistant Analysis System” on chest CT images and statistical analysis using SPSS. Their AI-based chest CT scan analysis was proven to be capable of identifying COVID-19 rapidly as well as accurately. On the other hand, Contreras et al. [116] analyzed the trends and errors of the COVID-19 pandemic using statistical-based approaches only. They initially defined random variables by modeling probability distribution functions followed by predictions using the ARIMA model. They have predicted the discharge rate by studying the cases, especially in Chile. Pandey et al. [117] analyzed COVID-19 outbreak data using Susceptible-Exposed-Infected-Removed (SEIR) and regression. Using both approaches, they predicted the cases of COVID-19 so that preventive measures could be taken on time. Based on RMSLE, SEIR was observed to be outperforming the regression model.

On the other hand, a prospective space-time scan statistic approach to observe the daily COVID-19 data has been utilized in [118, 119]. The authors therein analyzed the daily data by observing the characteristics of clusters at the country level. Sometimes it has been observed that there are chances of delay as well as errors in daily confirmed cases and epidemiological variables. Similarly, Sarkodie and Owusu [120] analyzed the relationship between COVID-19 cases and demises. Along with this relationship, they have analyzed the relationship between several other attributes in diagnosing disease spread. On the other hand, time-series data can forecast healthcare resource requirements by analyzing confirmed and recovered cases [121, 122]. A review of several mathematical and AI-based models of COVID-19 analysis is presented by Mohamadou et al. [123]. They have observed that most of the mathematical modeling related to COVID-19 analysis was based on two well-known methods, namely, SEIR and Susceptible-Infected-Recovered (SIR); meanwhile AI implementation was mainly based on CNNs using CXR and chest CT (CCT) samples. A survey of statistical approaches for analyzing the impacts of COVID-19 on global economy is presented by Verma et al. in [124].

## 6. Some Public Imaging Datasets for COVID-19 Research

Data collection is one of the essential steps towards the identification of any disease using deep-learning-based approaches. Generally, datasets of COVID-19 are categorized into two classes, namely, imaging data and statistical data, as shown in Figure 10.

As the name suggests, imaging data contains a chest CT scan and other radiographic images, that is, X-ray. Few such potential and famous imaging repositories for COVID-19 research are presented in Table 3. Few other datasets can be found in [125].

This type of data provides detailed insights into lung infections due to COVID-19, and the same can help in recognizing the disease. On the other hand, statistical data represents information like the total number of COVID-19 cases, total deaths, recovered cases, recovery rate, mortality rate, state, country-wise cases, and so forth. Most of the statistical data is about daily confirmed cases, which can be obtained from [102, 132, 133]. Mohamadou et al. [123] have also provided 24 datasets (mix of text, images, prevalence rate, etc.) that can also be used for detection and classification of COVID-19 research. Such type of data helps in calculating and predicting the COVID-19 outbreak. In a brief period, several repositories containing CT scan images and X-ray have been reported. However, every work related to deep learning presented in the preceding sections is based on either CT scan or X-ray images. Most of the datasets are growing day by day as per the availability of new data.

## 7. Discussion

For better understanding of the works done by several researchers on the fight with the COVID-19 outbreak, it is essential to present a comprehensive survey of their insights. It is clear from the several works presented in this study that researchers are encouraged by the potential of deep-learning-based approaches in fighting the COVID-19 pandemic. No doubt, deep learning has been successfully applied in solving various real-life problems. On the other hand, there are several pros and cons of using deep-learning-based approaches for solving problems. Some of them are pointed as follows.

### 7.1. Pros of Using Deep-Learning-Based Approaches

As compared to manual identification and recognition of diseases, deep learning provides several advantages if enough data is available for training. A few of the advantages are mentioned as follows:

1. Requiring less amount of time for screening patients after completion of training.
2. Providing the facility of automatic feature extraction even from unorganized data.
3. Learning from examples.
4. Higher accuracy as compared to manual examination.

### 7.2. Cons of Using Deep-Learning-Based Approaches

Despite several advantages, deep learning approaches also possess various limitations. A few of them are mentioned as follows:

1. Inability to distinguish between several types of pneumonia.
2. Lack of transparency and interpretability (sometimes it is hard to determine what imaging features are being used to determine output) [28].
3. The gap between the responses of lungs concerning different diseases. No method can present various types of lung infections and their diseases (also cannot impact of other parameters such as age, immune status, drug reactivity, smoking, etc.)
4. Deep-learning-based approaches generally expressing positivity or negativity of a disease but not able to predict the severity of a disease.
5. Challenging to predict the output based on low quality/contrast images.
6. Requiring a massive amount of data. Complex algorithms demand a high configuration of machines in CPU, Main Memory, dedicated GPU, and so forth.

### 7.3. Open Research Issues

It has been observed that in most of the works in which deep learning models and their variants were used, they were utilized mainly for binarized classification, that is, predicting the positivity and negativity of having COVID-19. Still, there exist several open research issues that need to be resolved over time:

1. Considering real-world data while predicting and forecasting the epidemic trends because it has been observed that most of the predictions models were unable to predict the actual trends of COVID-19.
2. Predicting the severity of disease using multiclass classification.
3. Reducing the healthcare burden, especially that on health workers, using AI-enabled approaches.
4. Predicting and forecasting mortalities, medical equipment, ICU/bed requirements, and other essential requirements.
5. Development of hybrid datasets with enriched epidemical characteristics.
6. Enhancing the prediction accuracies and deploying real-life solutions for coping with the COVID-19 outbreak.
7. Analysis of social media trends along with real-time data in predicting the COVID-19 outbreak.
8. Deploying AI-based postpandemic solutions that can minimize the impact and improve nations' economies.

## 8. Conclusion

The COVID-19 outbreak has affected almost all countries. For better prevention, timely diagnosis, social distancing, and isolation are the foremost requirements. Due to the rapid and exponential increment in COVID-19 cases, radiologists and hospitals are overburdened. Accurate and timely detection of 2019-nCoV is foremost required for reducing the burden on the healthcare sector. It is observed that AI-based examinations on CT scan and X-ray images are playing an essential role in diagnosing COVID-19. Nowadays, most of the radiologists are taking advantage of such approaches. The work embodied in this paper is focused on works done by several researchers using AI and deep-learning-based approaches for COVID-19 identification from two primary imaging modalities, that is, CT scan and X-ray. Most of the works reported for COVID-19 identification using deep learning approaches are based on the concept of transfer learning. However, a few of the researchers have developed their novel CNN architectures and claimed good accuracies. There is no doubt that deep-learning-based approaches save the potential amount of time in screening COVID-19 patients. However, diagnosing diseases from imaging data alone does not fulfill the minimum requirements. Thus, it is foremost required to combine these imaging diagnoses along with clinical observations for accurate and efficient diagnosis of COVID-19 so that we can try to minimize its outbreak. In the future, the task of automated COVID-19 identification may be extended towards severity identification and increasing the classification accuracies.

## Figures and Tables

**Figure 1:** (a) Sample X-ray images of COVID-19-affected lungs [2]. (b) Sample CT scan images of COVID-19 patients [3].

**Figure 2:** Relationship between NN, DL, ML, and AI.

**Figure 3:** DeepMind's protein structure prediction system [12].

**Figure 4:** The overall working of the AI4COVID-19 app [15] for distinguishing between a COVID cough and a non-COVID cough.

**Figure 5:** Sample confusion matrix.

**Figure 6:** The pipeline of operations performed in DeCoVNet [24].

**Figure 7:** Summary of COVID-19 image classification model [54].

**Figure 8:** Automatic identification of COVID-19 from chest X-ray images using DarkCovidNet [56].

**Figure 9:** Identification of COVID-19 from chest X-ray images using three existing models [58].

**Figure 10:** Classification of COVID-19 datasets.

**Table 1:** Performance analysis of several deep-learning-based models for diagnosis of COVID-19 from CT scan images.

Researchers	Deep learning model	Performance
Wang et al. [21]	Novel method (based on 3D U-Net++ [22] and ResNet50 [23])	0.99 AUC and 0.98 sensitivity
Zheng et al. [24]	DeCoVNet (based on U-Net [20])	90.1% accuracy
Song et al. [25]	DeepPneumonia	86% accuracy
Zhang et al. [26]	Novel method	92.49% accuracy
Li et al. [28]	COVNet (based on ResNet50 [23])	96% specificity and AUC of 0.96
Ardakani et al. [29]	Ten CNN models	99.51% accuracy using ResNet-101
Xu et al. [31]	Automated deep learning model (based on ResNet18)	86.7% accuracy
Chen et al. [32]	Deep learning model (based on U-Net++ [22])	98.85% accuracy
Shan et al. [33]	VB-Net (based on V-Net [34])	91.6% accuracy
Huang et al. [35]	Deep learning model (based on U-Net [20])	Quantification of CT parameters and analysis of lung opacities
Wang et al. [36]	Pretrained model	89.5% accuracy
Pathak et al. [37]	ResNet50 [23]	93% accuracy

**Table 2:** Performance analysis of several deep learning models for classification of COVID-19 from X-ray images.

Researchers	Deep learning model	Performance
Zhang et al. [45]	Novel	96% accuracy
Panwar et al. [46]	nCOVnet	97.62% accuracy
Stephen et al. [48]	Novel	95% accuracy
Wang and Wong [49]	Novel	83.5% accuracy
Ghosal and Tucker [57]	ResNet50V2	*ρ*=0.99
Toğaçar et al. [54]	MobileNetV2 and SqueezeNet	99.27% accuracy
Ozturk et al. [56]	DarkCovidNet (based on YOLO)	98.08% accuracy
Narin et al. [58]	ResNet50 [23], InceptionV3, and InceptionResNetV2	98% accuracy using ResNet50
Hemdan et al. [62]	VGG19, DenseNet201, MobileNetV2, Xception, ResNetV2, InceptionV3, and InceptionResNetV2	90% accuracy using VGG19
Sethy et al. [61]	Thirteen CNN models	95.38% accuracy using RestNet50
Khan et al. [64]	CoroNet (based on Xception)	89.6% accuracy
Rahimzadeh and Attar [65]	The concatenated network of Xception and ResNet50V2	99.50% accuracy
Chowdhury et al. [66]	DenseNet201, ResNet18, AlexNet, and SqueezeNet	98.3% accuracy using SqueezeNet
Apostolopoulos et al. [68]	VGG19, MobileNetV2, InceptionResNetV2, Inception, and Xception	98.75% accuracy using VGG19
Altan and Karasu [69]	EfficientNetB0	99.69% accuracy
Brunese et al. [70]	Transfer learning	97% accuracy
Ucar and Korkmaz [71]	Deep-SqueezeNet (based on SqueezeNet)	98.26% accuracy
Mahmud et al. [72]	CovXNet	97.4% accuracy

**Table 3:** Some COVID-19 public imaging repositories.

Contributor	Modality	Findings	Other details provided
Zhao et al. [3]	CT	COVID-19, non-COVID	Age, gender, medical history, severity, and other diseases
COVID-19 CT segmentation dataset [126]	CT	COVID-19	Ground-glass, consolidation, pleural effusion
Eduardo Soares et al. [127]	CT	COVID-19, normal	eXplainable deep neural network (xDNN)
Cohen et al. [2]	X-ray, CT	COVID-19, SARS, pneumonia, influenza, and other associated diseases.	Age, gender, survival, views
Italian Society of Medical and International Radiology [128]	X-ray, CT	COVID-19	Age, gender, other diseases, medical history
Radiological Society of North America [129]	X-ray, CT	COVID-19, pneumonia	Age, gender, CT findings
Wang et al. [130]	X-ray	COVID-19, pneumonia, normal	COVID-Net source code, age, gender, survival, views
Chowdhury et al. [66, 131]	X-ray	COVID-19, pneumonia, normal	Age, gender, survival, views

## Data Availability

All the data are shared in the main manuscript.
